The article "Correlation between Endometrial Vascular Endothelial Growth Factor Expression and Pregnancy Outcome of Frozen–Thawed Embryo Transfer in Patients with Repeated Implantation Failure" was retracted in 2023. Reasons: signs of a paper mill; suspected computer-generated content; unreliable results or conclusions; concerns about the data.

# Correlation between Endometrial Vascular Endothelial Growth Factor Expression and Pregnancy Outcome of Frozen–Thawed Embryo Transfer in Patients with Repeated Implantation Failure

**DOI:** 10.1155/2022/1937714

**Published:** 2022-09-29

**Authors:** Rui Jin, Wenye Ma, Dawei Tang, Fang Liu, Gang Bai, Mengmeng Reng

**Affiliations:** Medical Center, Yinchuan Maternal and Child Health Hospital, Yinchuan, Ningxia 750001, China

## Abstract

**Objective:**

Vascular endothelial growth factor (VEGF) is a well-known angiogenic factor that is essential to numerous physiological and pathological processes. VEGF also contributes to embryo implantation by promoting embryo development, enhancing endometrial receptivity (ER), and promoting interactions between the endometrium and developing embryo. Changes in VEGF expression are linked to repeated implantation failure (RIF). Control endometrial tissues demonstrated an increase in VEGF expression during the implant window period, which promoted early villous vascularization and embryo implantation. The purpose of this study is to investigate the relationship between RIF and the expression of ER markers, such as VEGF during the implantation window stage.

**Methods:**

The Yinchuan Maternal and Child Health Hospital collected 192 cases of FET endometrial tissues in the implantation window stage between January 2019 and December 2021. Immunohistochemistry was utilized to measure the levels of VEGF expression in patients with RIF (RIF group, *n* = 82) and patients with a successful pregnancy (control group, *n* = 110). The relationship between VEGF and the RIF group was analyzed using Spearman's correlation coefficient.

**Results:**

VEGF levels were significantly lower during the implantation window stage (*P* < 0.05).

**Conclusion:**

VEGF was expressed in planting window stage. The decrease of VEGF during the implantation window was correlated with RIF.

## 1. Introduction

Repeated implantation failure (RIF) is one of the most significant obstacles in human reproduction. Because of the fact that RIF was initially regarded as a relatively heterogeneous entity, it was challenging to establish a definition. Due to the variety of RIF definitions, data on RIF incidence are rather limited [1]. Implantation failures are thought to be due to either defective embryo quality or endometrial receptivity (ER) [2]. Although a number of factors associated with these clinical entities have been recognized, in the majority of cases the underlying factors and mechanisms are unknown, and consequently treatment options are limited [3].

The mechanism behind embryo implantation is complicated; the two most crucial factors for an effective embryo implantation are a good ER and high-quality embryo. Many recent clinical randomized controlled studies and meta-analyses have found that endometrial stimulation aids embryo implantation and greatly enhances the pregnancy rate in instances of artificial insemination, frozen–thawed embryo transfer (FET) cycles, recurrent miscarriage, and previous transplant failure. Endometrial stimulation may increase the production of implantation-related local factors, such as transforming growth factor, homeobox protein, and interleukins, and enhance ER, thereby enhancing pregnancy outcomes [4].

The article "Correlation between Endometrial Vascular Endothelial Growth Factor Expression and Pregnancy Outcome of Frozen–Thawed Embryo Transfer in Patients with Repeated Implantation Failure" was retracted in 2023. Reasons: signs of a paper mill; suspected computer-generated content; unreliable results or conclusions; concerns about the data.

Vascular endothelial growth factor (VEGF) is an endothelial cell-specific mitogen in vitro that is known to be the key factor responsible for vasculogenesis and angiogenesis in a variety of models [5]. VEGF also contributes to embryo implantation by promoting embryo development, enhancing ER, and promoting interactions between the endometrium and developing embryo. Changes in VEGF expression have been linked to RIF [6, 7]. As one of the biological markers used to evaluate ER, VEGF can aid in vascularization tolerance for implantation.

The technology of FET has been around for the past 40 years. During this time, the clinical pregnancy rate has remained between 50 and 60%, while the embryo implantation rate has remained between 30 and 40%. Improving the pregnancy rate of patients with non-embryonic factors is highly reliant on the ability to enhance ER. In this study, 192 cycles of luteum endometrial tissue from the Yinchuan Maternal and Child Health Care Reproductive Center were used to implement freeze–thaw embryo transfers, including 82 cases of RIF and 112 cases of patients experiencing their first transplant pregnancy. Immunohistochemical analysis of endometrial VEGF expression was used to examine the expression of related factors and RIF for the clinical study of the pathogenesis of RIF and to provide experimental research clues.

## 2. Data and Methods

### 2.1. Subject Investigated

From January 2019 to December 2021, the patients were between the ages of 25 and 39 years, with 82 cycles in the study group consisting of patients who had undergone embryo transplantation more than three times, and 112 cycles consisting of patients who had their first successful pregnancy. All of the embryos transplanted were of high quality. Exclusion criteria for the study included endometriosis, uterine fibroids, adenomyosis, hydrofallopian duct, polycystic ovary syndrome, abnormal uterine structures, poor lining or morphology, hypercoagulability or easy thrombosis, no prior history of ovarian surgery, and the absence of hormonal or hormone therapy and uterine procedures within the previous three months. This study was approved by the hospital's ethics committee, and each participant provided informed consent.

The article "Correlation between Endometrial Vascular Endothelial Growth Factor Expression and Pregnancy Outcome of Frozen–Thawed Embryo Transfer in Patients with Repeated Implantation Failure" was retracted in 2023. Reasons: signs of a paper mill; suspected computer-generated content; unreliable results or conclusions; concerns about the data.

### 2.2. Research Technique

#### 2.2.1. Endometrial Collection

The patient's endometrial tissue was removed on the seventh day following the preparatory ovulation cycle in order to prepare it for freezing and freeze–thaw embryo transfer. It was then immersed in 4% formaldehyde, fixed for no longer than 24 hours for immunohistochemical analysis, and then embedded in paraffin. The other portion was stored in a −80°C refrigerator for immunohistochemistry analysis.

#### 2.2.2. Evaluation Criteria for Immunohistochemical Results

Random selection was used to choose five high magnification fields (400 times) for each stained piece. The phosphatase buffer reagent was used in place of the primary antibody as a negative control, and the sections were read without the use of any specific negative coloring of the images. The staining results of positive cells need to fulfil the following conditions: the tissue cell structure must be complete and distinct; the staining of positive cells must be significantly more intense than the background; and the positioning of positive particles must be evidently distinct. According to the intensity of staining of brown particles in the cytoplasm, no cells have any staining (−), positive staining of cells below 25% was recorded as weak positive (+), positive staining of 25–50% cells was recorded as positive staining of medium intensity (+ +), and positive staining of 50% cells was recorded as strong positive (+ + +).

#### 2.2.3. Observation Indicators

General condition, endometrial thickness, morphology, embryo score, and pregnancy outcome of the two patient groups were included as observation indicators.

### 2.3. Statistical Analysis

The SPSS19.0 Windows statistical software was used to analyze the collected data. The *t*-test was utilized for the analysis of measurement data, while the *χ*^2^test was employed for the analysis of count data. *P* < 0.05 indicated a statistically significant difference.

## 3. Results

### 3.1. Basic Information of the Patients in Both Groups

In this study, 192 patients were evaluated during the implant window period, and age, infertility years, and endometrial thickness were compared between the two groups.  Table 1 summarizes the comparison of basic information between the two patient groups.

### 3.2. Comparison of VEGF Positive Expression in the Planting Window between the Two Groups

VEGF, insulin-like growth factor, and leukemia inhibitory factor were detected in the implant window of both groups. However, the expression of patients in the RIF group was significantly lower than that of patients in the control group.  Table 2 show the endometrial VEGF expression comparison between the two patient groups.

The article "Correlation between Endometrial Vascular Endothelial Growth Factor Expression and Pregnancy Outcome of Frozen–Thawed Embryo Transfer in Patients with Repeated Implantation Failure" was retracted in 2023. Reasons: signs of a paper mill; suspected computer-generated content; unreliable results or conclusions; concerns about the data.

## 4. Discussion

The term “endometrial receptivity” describes the unique time frame during which the endometrium is “receiving” the embryo implant, also known as the “implant window period” (window of implantation) of the endometrium. Typically, during this time, the endometrial morphology, tissue structure, and proteins undergo a series of secreted changes [8]. Embryos are only implanted during this time, and implantation fails either before or after the planting window opens. Currently, the endometrium's tolerance is primarily assessed through ultrasound examination of blood flow, thickness, and morphology [9]. The expression of various endometrial factors is increasingly regarded as a valuable method for determining ER. The analysis of the expression of various factors in the endometrium during the endometrial implantation window period can objectively reflect the state of the endometrium, provide a clinical basis for embryo transfer time, and effectively promote the improvement of the embryo implantation rate [10]. VEGF can act on both the endometrium and the embryo [11]. The expression of the three factors increases gradually during the female luteal corpus stage and reaches a peak during the implant window stage, which is closely associated with the formation of ER [12]. It is positively correlated with endometrial acceptance of the embryo, a critical factor for embryo implantation and pregnancy success [13]. As one of the biological markers used to evaluate ER, VEGF can facilitate vascularization tolerance for implantation [14, 15]. During the implant window period, control endometrial tissues exhibited an increase in VEGF expression, which facilitated embryonic implantation and early villous vascularization [16, 17]. The positive endometrial VEGF expression of the RIF group was significantly lower than that of the control group, and its reduced positive expression may be associated with the decrease in subendometrial blood perfusion, which affects the ER, ultimately results in the failure of embryo implantation, and then causes infertility.

## 5. Conclusion

In this study, the immunohistochemical technique was used to determine the endometrial VEGF localization and expression during the embryo planting window for patients who had undergone a freeze–thaw embryo transplant during the preparatory period. There are relatively few cases, but the researchers are optimistic that multi-center studies in the future will be able to predict endometrial tolerance, facilitate embryo implantation, and increase the pregnancy rate.

The article "Correlation between Endometrial Vascular Endothelial Growth Factor Expression and Pregnancy Outcome of Frozen–Thawed Embryo Transfer in Patients with Repeated Implantation Failure" was retracted in 2023. Reasons: signs of a paper mill; suspected computer-generated content; unreliable results or conclusions; concerns about the data.

## Figures and Tables

**Table 1:** Comparison of basic information between the two patient groups.

Group	*n* (example)	Age (year)	Infertility years (years)	Inner membrane thickness (mm)
RIF group	82	32.74 ± 2.07	0.045 ± 3.00	0.729 ± 1.75
Control group	110	32.80 ± 2.09	0.704 ± 2.79	9.87 ± 1.68
*T*-value		−0.166	0.711	−0.544
*P*-value		0.868	0.478	0.588

**Table 2:** Comparison of endometrial VEGF expression between the two patient groups.

Group	*N*	Positive expression of VEGF
RIF group	82	40.24% (33/82)
Control group	110	17.14% (12/70)
*χ* ^2^		9.67
*P*-value		0.002

## Data Availability

Data supporting this research article are available from the corresponding author or first author on reasonable request.
